# TSM-Based Adaptive Fuzzy Control of Robotic Manipulators with Output Constraints

**DOI:** 10.1155/2021/5812584

**Published:** 2021-07-13

**Authors:** Fei Yan, Shubo Wang

**Affiliations:** ^1^School of Automation, Qingdao University, Qingdao 266071, China; ^2^Shandong Key Laboratory of Industrial Control Technology, Qingdao 266071, China

## Abstract

This paper proposes an adaptive control scheme based on terminal sliding mode (TSM) for robotic manipulators with output constraints and unknown disturbances. The fuzzy logic system (FLS) is developed to approximate unknown dynamics of robotic manipulators. An error transformation technique is used in the process of controller design to ensure that the output constraints are not violated. The advantage of the error transformation compared to traditional barrier Lyapunov functions (BLFs) is that there is no need to design a virtual controller. Thus, the design complexity of the controller is reduced. Through Lyapunov stability analysis, the system state can be proved to converge to the neighborhood near the balanced point in finite time. Extensive simulation results illustrated the validity of the proposed controller.

## 1. Introduction

In recent decades, robotic manipulators have been widely used in industrial and aerospace fields due to the rapid development of artificial intelligence [1–6]. As the model uncertainty, input, and measurement disturbance always exist, some linear control schemes cannot obtain satisfactory performance. Therefore, many researchers utilize adaptive control [7–11], robust control [12, 13], output-feedback control [14, 15], and learning control strategies [16, 17] to overcome above difficulties. The security issues caused by output constraints cannot be ignored because humans interact with robotic manipulators.

To handle the problem of output constraints, many techniques have been developed [18–21]. In [22], a robust adaptive neural network (NN) control is utilized to guarantee the prescribed performance of the multiple-input multiple-output (MIMO) systems. In [23], a barrier Lyapunov function is used to guarantee the output constraints, which provides more flexibility and reduces the requirements for prerequisites. For nonlinear system, an optimal control strategy which transforms the constrained system into a novel one without output constraints is proposed in [24]. In [25], an adaptive neural network tracking control is proposed for robotic manipulators subjected to output constraints. The output constraints of some systems are not immutable; thus, to handle this problem, an asymmetric barrier Lyapunov function is used in the design process of the controller in [26]. Recently, a new robust control is developed in [27]. This control method first converts the output constraints into the error constraints. Then, an error transformation technique is employed, which changes the constrained error system into an unconstrained system.

Intelligent controls have been widely used to cope with model uncertainty due to their approximation ability. According to combine fuzzy system or neural network with adaptive control, online parameters estimation can be realized, which improves the feasibility of the control scheme [28–34]. A novel adaptive fuzzy controller is presented to guarantee the stability of closed-loop system in [35]. For a class of uncertain MIMO nonlinear systems in the discrete-time form, a control strategy that uses higher order neural networks to approximate the desired controllers is proposed in [36]. An adaptive neural network scheme considering unknown output hysteresis is studied in [37], which used only two learning parameters so that the computational burden is greatly reduced. In [25], two neural networks are utilized in the controller: one is used to approximate the unknown dynamic model, and the other is used to approximate the error of the input dead zone.

Sliding mode control (SMC) is widely used in motion control, because of its simple algorithm and good robustness [38]. With the development of sliding mode control technology, there are many new sliding mode control schemes. In [39], a radial basis function (RBF) neural network sliding mode control scheme is used to realize the asymptotic stability of rigid robotic manipulators, in which RBF neural network is used to estimate unknown dynamics. An integral sliding mode adaptive control scheme is proposed to realize system signals uniformly ultimately bounded in [40]. A second-order sliding mode control algorithm is presented in [41]. Fast terminal sliding mode control schemes are used to control the single input single output system (SISO) and the robotic manipulators, respectively, in [42, 43]. Both have achieved fast and high-precision tracking performance. For dual-inertia driving systems, an adaptive control scheme combining sliding mode with prescribed performance function is proposed in [44]. There are many papers that use terminal sliding mode to control the manipulators, but few researches on the manipulators with output constrains and model uncertainty are carried out. And most of the existing methods to solve the problem of output constrains are using barrier Lyapunov function. These methods need to design additional virtual controllers, which will increase the complexity of the controller.

To better solve the trajectory tracking problem of a class of manipulators with output constrains and model uncertainty, a novel adaptive fuzzy control scheme that combines error transformation with finite time sliding surface is designed. Using the fuzzy logic system to approximate model uncertainty can improve tracking performance. The problem of output constraints is solved by introducing an error transformation function. This error transformation function changes the output constraints into the error constrains. Therefore, not only can it be ensured that the output constraints are not violated, but also the transient response can be improved. The error after conversion is used in the sliding mode surface, and the convergence of the system is proved by the Lyapunov stability theorem. The main contributions are summarized as follows:

1. To prevent the contravention of output constraints, the error transformation is used in the controller design. The introduction of virtual controller is avoided which reduces the cost of calculation. At the same time, the effect of transient response is improved.
2. Modify the sliding mode surface. The transformed error is applied to the sliding surface, which guarantees that system output constraints not only are not violated but also achieve the steady-state error converge to near the balanced point in finite time.

In what follows, first, the dynamic model, fuzzy logic system, and error transformation are presented, followed by the derivation of the controller. Then, the stability analysis and mathematical proof are given. The paper ends with some comparative simulations and conclusions.

## 2. Problem Formulation and Preliminaries

### 2.1. Dynamic Model of the Robotic Manipulator

An *n*-degree-of-freedom robotic manipulator with unknown disturbance can be described as

(1) $$\begin{array}{c} M\left(q\right)\ddot{q}+C\left(q,\dot{q}\right)\dot{q}+G\left(q\right)=\tau +\tau_{d}, \end{array}$$

where *M*(*q*) denotes the symmetric positive definite inertia matrix, $C\left(q,\dot{q}\right)$ represents the Coriolis/centripetal torque, *G*(*q*) is the gravity torque, *τ*_*d*_ denotes the unknown external disturbances, *τ* is the control input torque, and *q* is the angular position.

**Property 1 (see [25]).**

The matrix *M*(*q*) is positive definite symmetric matrix.

**Property 2 (see [25]).**

The matrix $\dot{M}-2C\left(q,\dot{q}\right)$ is skew-symmetric.

In practice, due to modeling error, physical parameter perturbation, and other factors, the system model always has uncertainty; thus, the following formula holds:

(2) $$\begin{array}{c} M=M_{0}+M_{n},\\ C=C_{0}+C_{n},\\ G=G_{0}+G_{n}, \end{array}$$

where *M*_0_, *C*_0_,  and *G*_0_ denote the nominal part of the model and *M*_*n*_, *C*_*n*_, and *G*_*n*_ denote the mode uncertainty.

The control problem is to design a control law to ensure the system output state *q* can track the desired *q*_*d*_ and to guarantee the constraints are not violated simultaneously. In order to verify the feasibility of proposed control scheme, the following assumptions are given.

**Assumption 1 (see [27]).**

For every desired trajectory *q*_*d*_*i*__, the inequality $-{\underline{k}}_{d_{i}}\leq q_{d_{i}}\leq {\bar{k}}_{d_{i}}$ is held, where positive constants ${\underline{k}}_{d_{i}},{\bar{k}}_{d_{i}}$ denote the lower and upper bound, respectively. There exists positive constant *k*_*d*_*i*__^*∗*^ satisfying $\max\left\{{\underline{k}}_{d_{i}},{\bar{k}}_{d_{i}}\right\}\leq k_{d_{i}}^{*}<k_{o_{i}}$ for any *k*_*o*_*i*__ > 0.

**Assumption 2 (see [45]).**

The disturbance *τ*_*d*_ is bounded such that $\tau_{d}\leq \bar{\tau }$ holds for positive constants $\bar{\tau }$.

**Assumption 3 (see [46]).**

The reference trajectory *q*_*d*_ and its first two time derivatives ${\dot{q}}_{d},{\ddot{q}}_{d}$ are bounded. Moreover, the angular position *q* and speed $\dot{q}$ are measurable.

### 2.2. Fuzzy Logic Systems

The fuzzy system can be used to approximate unknown nonlinear function due to their universal approximation ability. The advantage of fuzzy system is that it can use linguistic information effectively [47]. The structure of fuzzy system is shown in Figure 1. The design steps of fuzzy system are as follows [16]:

1. Define *N*_*i*_ fuzzy sets for each variable *x*_*i*_.
2. Set ∂=∏_*i*=1_^*n*^*N*_*i*_ fuzzy IF-THEN rules: if *x*_1_ is *A*_1_^*k*_1_^ and … and *x*_*n*_ is *A*_1_^*k*_*n*_^; then *y* is *W*^*k*_1_*k*_2_^, where *k*_*i*_=1,2,…, *N*_*i*_, *i*=1,…, *n*.
3. Using the fuzzy inference engine and the defuzzifier, the fuzzy system can be obtained as

(3) $$\begin{array}{c} \hat{f}=\frac{\sum_{k=1}^{l}y_{k}\left(\prod_{i=1}^{n}\mu_{A_{i}^{k}}\left(x_{i}\right)\right)}{\sum_{k=1}^{l}\left(\prod_{i=1}^{n}\mu_{A_{i}^{k}}\left(x_{i}\right)\right)}, \end{array}$$

with *μ*_*A*_*i*_^*k*^_(*x*_*i*_)=exp[−((*x*_*i*_ − *c*_*ik*_)^2^/2*b*_*ik*_^2^)], where *μ*_*A*_*i*_^*k*^_(*x*_*i*_) denotes the Gaussian membership function. *c*_*ik*_ and *b*_*ik*_ denote the center and the width of the Gaussian function, respectively.

For clarity, we now arrange (3) into the following form:

(4) $$\begin{array}{c} \hat{f}=\hat{\Theta }\Phi \left(x\right), \end{array}$$

where $\hat{\Theta }={\left[y_{1},\ldots ,y_{l}\right]}^{T}$ is the free parameters and Φ(*x*) is given as

(5) $$\begin{array}{c} \Phi \left(x\right)=\frac{\prod_{i=1}^{n}\mu_{A_{i}^{k}}\left(x_{i}\right)}{\sum_{k=1}^{l}\left(\prod_{i=1}^{n}\mu_{A_{i}^{k}}\left(x_{i}\right)\right)}. \end{array}$$

Therefore, a nonlinear function can be expressed as

(6) $$\begin{array}{c} f=\hat{\Theta }\Phi \left(x\right)+\varepsilon , \end{array}$$

where *ε* is the approximation error which satisfies $\left\|\varepsilon \right\|\leq \left\|\bar{\varepsilon }\right\|$; $\bar{\varepsilon }$ is a positive constant.

### 2.3. Error Transformation

To realize the control goal, we first define the tracking error as

(7) $$\begin{array}{c} e_{1}=q-q_{d}, \end{array}$$

where *q*=[*q*_1_,…, *q*_*i*_,…, *q*_*n*_], *i*=1,…, *n*, denotes the position vector of each joint, *q*_*d*_=[*q*_*d*_1__,…, *q*_*d*_*i*__,…, *q*_*d*_*n*__] denotes the target trajectory, and *e*_1_ can be expressed as [*e*_11_, *e*_12_,…, *e*_1*n*_].

**Lemma 1 (see [27]).**

Consider an Euler-Lagrange system. If the initial error satisfies *e*_*i*_(0) < *k*_*b*_*i*__, ∀*i*=1,…, *n* and the transformed error variables are bounded, then the closed-loop error is bounded and the output of system *x*_1*i*_ remains bounded by the imposed output constraints, e.g., |*x*_1*i*_| < *k*_*o*_*i*__, ∀*i*=1,…, *n*.

To ensure the constraints are not violated, we use an error transformation as [27]. This method changes the output constraints into error constraints and it can be expressed as

(8) $$\begin{array}{c} k_{b_{i}}=k_{o_{i}}-k_{d_{i}}^{*}, \end{array}$$

where *k*_*d*_*i*__^*∗*^ is defined in assumption 1, *k*_*o*_*i*__ are the output constraints of the output *q*_*i*_, and *k*_*b*_*i*__ are the error constraints. They are shown in Figure 2.

For the next stability analysis, the error transformation variable *z*_1_ is defined as

(9) $$\begin{array}{c} z_{1}={\dot{e}}_{1}+P_{1}\left(e_{1}\right)e_{1}, \end{array}$$

where *P*_1_(*e*_1_) is a symmetric diagonal matrix, defined as

(10) $$\begin{array}{c} \left[\begin{array}{ccc} \frac{p_{1}}{\left(k_{b_{1}}^{2}-e_{11}^{2}\right)} & \ldots & 0\\ \vdots & \frac{p_{i}}{\left(k_{b_{i}}^{2}-e_{1i}^{2}\right)} & \vdots \\ 0 & \cdots & \frac{p_{n}}{\left(k_{b_{n}}^{2}-e_{1n}^{2}\right)} \end{array}\right],\;i=1,\ldots ,n, \end{array}$$

where *p*_*i*_ are positive constants that we need to design. *e*_1_*i*__ are the tracking errors on *i*^th^ robot joint and defined in (7).

The time derivative of *z*_1_ in (9) can be calculated as

(11) $$\begin{array}{c} {\dot{z}}_{1}={\ddot{e}}_{1}+{\dot{P}}_{1}\left(e_{1}\right)e_{1}+P_{1}\left(e_{1}\right){\dot{e}}_{1}\\ ={\ddot{e}}_{1}+\text{diag}\left[\frac{2p_{i}e_{i}^{2}}{{\left(k_{b_{i}}^{2}-e_{i}^{2}\right)}^{2}}\right]{\dot{e}}_{1}+\text{diag}\left[\frac{p_{i}}{k_{b_{i}}^{2}-e_{i}^{2}}\right]{\dot{e}}_{1}\\ ={\ddot{e}}_{1}+P_{2}\left(e_{1}\right){\dot{e}}_{1}, \end{array}$$

where *P*_2_(*e*_1_) is a symmetric diagonal matrix, which is obtained by extracting common factors from the two rightmost items in (11) and can be expressed as

(12) $$\begin{array}{c} \left[\begin{array}{ccc} \frac{p_{1}\left(k_{b_{1}}^{2}+e_{11}^{2}\right)}{{\left(k_{b_{1}}^{2}-e_{11}^{2}\right)}^{2}} & \ldots & 0\\ \vdots & \frac{p_{i}\left(k_{b_{i}}^{2}+e_{1i}^{2}\right)}{{\left(k_{b_{i}}^{2}-e_{1i}^{2}\right)}^{2}} & \vdots \\ 0 & \cdots & \frac{p_{n}\left(k_{b_{n}}^{2}+e_{1n}^{2}\right)}{{\left(k_{b_{n}}^{2}-e_{1n}^{2}\right)}^{2}} \end{array}\right],\;i=1,\ldots ,n. \end{array}$$

## 3. Controller Design

According to the above conversion of errors, the original system with output constraints is transformed into an unconstrained system. By Lemma 1, we just need to design a controller to ensure the variable *z*_1_ is bounded so that the system can track the desired trajectory and the output constraints are not violated. The control structure is shown in Figure 3.

A terminal sliding mode variable is defined as

(13) $$\begin{array}{c} r=z_{1}+k_{1}{\text{sig}}^{a_{2}}e_{1}={\dot{e}}_{1}+P_{1}\left(e_{1}\right)e_{1}+k_{1}{\text{sig}}^{a_{2}}e_{1}, \end{array}$$

where *k*_1_ is a positive constant. *a*_2_=(*p*/*q*) is satisfied *p* < *q* and *p* and *q* are coprime positive odd numbers. sig^*a*^(·)=|·|^*a*^sgn(·), and sgn(·) denotes the signum function.

Differentiating (13), we can get

(14) $$\begin{array}{c} \dot{r}={\ddot{e}}_{1}+P_{2}\left(e_{1}\right){\dot{e}}_{1}+k_{1}a_{2}{\left|e_{1}\right|}^{a_{2}-1}{\dot{e}}_{1}. \end{array}$$

Multiplying (14) by *M*_0_(*q*), one has

(15) $$\begin{array}{c} M_{0}\dot{r}=\left(M_{0}+M_{n}\right){\ddot{e}}_{1}-M_{n}{\ddot{e}}_{1}+M_{0}P_{2}\left(e_{1}\right){\dot{e}}_{1}+M_{0}k_{1}a_{2}{\left|e_{1}\right|}^{a_{2}-1}{\dot{e}}_{1}\\ =\tau +\tau_{d}-C\left(q,\dot{q}\right)\dot{q}-G\left(q\right)-M{\ddot{q}}_{d}-M_{n}{\ddot{e}}_{1}+M_{0}P_{2}\left(e_{1}\right){\dot{e}}_{1}+M_{0}k_{1}a_{2}{\left|e_{1}\right|}^{a_{2}-1}{\dot{e}}_{1}\\ =\tau +\tau_{d}-C\left(q,\dot{q}\right)r+C\left(q,\dot{q}\right)r-C\left(q,\dot{q}\right)\dot{q}-G\left(q\right)\\ -M{\ddot{q}}_{d}-M_{n}{\ddot{e}}_{1}+M_{0}P_{2}\left(e_{1}\right){\dot{e}}_{1}+M_{0}k_{1}a_{2}{\left|e_{1}\right|}^{a_{2}-1}{\dot{e}}_{1}\\ =\tau +\tau_{d}-C_{0}\left(q,\dot{q}\right)r-C_{n}\left(q,\dot{q}\right)r+C\left(q,\dot{q}\right)r-C\left(q,\dot{q}\right)\dot{q}\\ -G\left(q\right)-M{\ddot{q}}_{d}-M_{n}{\ddot{e}}_{1}+M_{0}P_{2}\left(e_{1}\right){\dot{e}}_{1}+M_{0}k_{1}a_{2}{\left|e_{1}\right|}^{a_{2}-1}{\dot{e}}_{1}\\ =\tau +\tau_{d}-C_{0}\left(q,\dot{q}\right)r+M_{0}P_{2}\left(e_{1}\right){\dot{e}}_{1}+M_{0}k_{1}a_{2}{\left|e_{1}\right|}^{a_{2}-1}{\dot{e}}_{1}-F\left(q,\dot{q},{\ddot{q}}_{d},{\dot{e}}_{1},{\dot{e}}_{1}\right), \end{array}$$

where $F\left(q,\dot{q},{\ddot{q}}_{d},e_{1},{\dot{e}}_{1}\right)=M{\ddot{q}}_{d}+M_{n}{\ddot{e}}_{1}+G\left(q\right)+C\left(q,\dot{q}\right)\dot{q}-C\left(q,\dot{q}\right)r$ is the unknown dynamics. The nonlinear dynamics function $F\left(q,\dot{q},{\ddot{q}}_{d},e_{1},{\dot{e}}_{1}\right)$ is continuous and thus it can be approximated by a FLS as

(16) $$\begin{array}{c} \Theta \Phi \left(Z\right)=F\left(q,\dot{q},{\ddot{q}}_{d},e_{1},{\dot{e}}_{1}\right)+\varepsilon , \end{array}$$

where Θ is the optimal constant parameter vector. Φ(·) is the fuzzy basis function. $Z=\left[q,\dot{q},{\ddot{q}}_{d},e_{1},{\dot{e}}_{1}\right]$ is the input vector. *ε* is the approximation error of the FLS, which satisfies $\left\|\varepsilon \right\|\leq \left\|\bar{\varepsilon }\right\|$.

Then, substituting (16) into (15), the open-loop error system can be obtained as

(17) $$\begin{array}{c} M_{0}\dot{r}=\tau +\tau_{d}-C_{0}\left(q,\dot{q}\right)r+M_{0}P_{2}\left(e_{1}\right){\dot{e}}_{1}\\ +M_{0}k_{1}a_{2}{\left|e_{1}\right|}^{a_{2}-1}{\dot{e}}_{1}-\Theta \Phi \left(Z\right)+\varepsilon . \end{array}$$

The optimal parameter vector Θ cannot be obtained in practice. Thus, the estimation $\hat{\Theta }$ replaces Θ in the process of designing the controller. Thus, the estimation of the nonlinear function can be expressed as

(18) $$\begin{array}{c} \hat{F}\left(q,\dot{q},{\ddot{q}}_{d},e_{1},{\dot{e}}_{1}\right)=\hat{\Theta }\Phi \left(Z\right). \end{array}$$

The fuzzy system parameter $\hat{\Theta }$ can be updated by the following adaptive law:

(19) $$\begin{array}{c} \dot{\hat{\Theta }}=-\Gamma \left[\Phi \left(Z\right)r+\sigma \hat{\Theta }\right], \end{array}$$

where Γ is a positive gain matrix and *σ* denotes the forgetting factor.

**Remark 1 .**

The adjustment of learning gain Γ needs to balance rapidity and stability. A large Γ will improve the adaptation speed, but will lead to high-frequency oscillations in the control response. Conversely, a small Γ will suppress high-frequency oscillations, but will reduce the adaptation speed. The forgetting factor is a positive constant, which is usually chosen as a small value. The role of forgetting factor is to improve the robustness to bounded disturbance and to accelerate the adaption speed.

A TSM-based controller is designed to obtain the convergence of system state. Based on (17) and subsequent stability analysis, the control law *τ* is designed as

(20) $$\begin{array}{c} \tau =-kr-M_{0}P_{2}\left(e_{1}\right){\dot{e}}_{1}-M_{0}k_{1}a_{2}{\left|e_{1}\right|}^{a_{2}-1}{\dot{e}}_{1}+\hat{\Theta }\Phi \left(Z\right)-\beta {\text{sig}}^{r_{2}}r, \end{array}$$

where *k* and *β* are positive constants that designed by designer. *r*_2_=(*m*/*n*) is satisfied *m* < *n* and *m* and *n* are coprime positive odd numbers.

Substituting (20) into (17), the closed-loop tracking error system can be obtained as

(21) $$\begin{array}{c} M_{0}\dot{r}=-kr+\tau_{d}-C_{0}\left(q,\dot{q}\right)r+\tilde{\Theta }\Phi \left(Z\right)+\varepsilon -\beta {\text{sig}}^{r_{2}}r, \end{array}$$

where $\tilde{\Theta }$ is the error between ideal value and estimated value.

**Remark 2 .**

Contrary to conventional TSM control scheme, e.g., [46], the error transformation is used in the controller to prevent the contravention of output constraints. This error transformation technique changes the output constraints into error constraints. Consequently, the transient response is improved. Compared with barrier Lyapunov function, the advantage of error transformation is that the virtual variables are not designed.

### 3.1. Stability Analysis

**Lemma 2 (see [48]).**

If a Lyapunov function *V*(*x*) is bounded and its derivative $\dot{V}\left(x\right)\leq -\lambda V\left(x\right)+C$, where *λ* and *C* are positive constants, then the solution *x* is bounded.

**Lemma 3 (see [43]).**

For a second-order system like (1), if there is a positive definite function *V*(*x*) and parameters *λ*_1_, *λ*_2_ > 0, 0 < *γ* < 1, *v* ≥ 0 satisfies the following inequality:

(22) $$\begin{array}{c} \dot{V}\left(x\right)+\lambda_{1}V\left(x\right)+\lambda_{2}V^{\gamma }\left(x\right)\leq v, \end{array}$$

then the system state can converge to the compact set Ω, defined by

(23) $$\begin{array}{c} \Omega ≔\left\{x|V\left(x\right)\leq \min\left\{\frac{v}{\lambda_{1}},{\left(\frac{v}{\lambda_{2}}\right)}^{\left(1/\gamma \right)}\right\}\right\}, \end{array}$$

and the upper bound of convergence time *T* satisfies

(24) $$\begin{array}{c} T=\frac{1}{\lambda_{1}\left(1-\gamma \right)}\ln\frac{\lambda_{1}V^{1-\gamma }\left(x_{0}\right)+\lambda_{2}}{\lambda_{2}}. \end{array}$$

The main conclusions of this paper can be summarized as follows.

**Theorem 1 .**

Consider robotic dynamic system (1), with bounded assumptions and initial conditions; TSM-based adaptive fuzzy controller is given as (20), as well as adaptive law (19):

1. The closed-loop system is ultimately uniformly bounded and the output constraints are not violated
2. The tracking error *e*_1_ converges to neighborhood near the zero point in finite time

**Proof**

1. A positive definite Lyapunov function is chosen as

(25) $$\begin{array}{c} V_{1}=\frac{1}{2}rM_{0}r+\frac{1}{2}\tilde{\Theta }\Gamma^{-1}\tilde{\Theta }. \end{array}$$

The time derivative of (25) is

(26) $$\begin{array}{c} {\dot{V}}_{1}=rM_{0}\dot{r}+\frac{1}{2}r{\dot{M}}_{0}r+\tilde{\Theta }\Gamma^{-1}\dot{\tilde{\Theta }}\\ =-kr^{2}-\beta {\left|r\right|}^{r_{2}}r\mathrm{sgn}\left(r\right)+r\tau_{d}+r\varepsilon \\ +r\tilde{\Theta }\Phi \left(Z\right)-r\tilde{\Theta }\Phi \left(Z\right)-\sigma {\tilde{\Theta }}^{T}\hat{\Theta }, \end{array}$$

where (19) and (21) are used.

According to average value inequality, we can get

(27) $$\begin{array}{c} r\tau_{d}+r\varepsilon \leq r^{2}+\frac{1}{2}\tau_{d}^{2}+\frac{1}{2}\varepsilon^{2}\leq r^{2}+\frac{1}{2}\tau_{d}^{2}+\frac{1}{2}{\bar{\varepsilon }}^{2}. \end{array}$$

Since$-{\tilde{\Theta }}^{T}\hat{\Theta }=-{\tilde{\Theta }}^{T}\left(\Theta +\tilde{\Theta }\right)=-{\tilde{\Theta }}^{T}\tilde{\Theta }-{\tilde{\Theta }}^{T}\Theta$ and $-{\tilde{\Theta }}^{T}\Theta \leq \left(1/2\right){\tilde{\Theta }}^{T}\tilde{\Theta }+\left(1/2\right)\Theta^{T}\Theta$, it simply implies

(28) $$\begin{array}{c} -{\tilde{\Theta }}^{T}\hat{\Theta }\leq -\frac{1}{2}{\tilde{\Theta }}^{T}\tilde{\Theta }+\frac{1}{2}\Theta^{T}\Theta . \end{array}$$

Substituting (27) and (28) into (26), we can obtain

(29) $$\begin{array}{c} {\dot{V}}_{1}\leq -\left(k-I\right)r^{2}-\beta {\left|r^{2}\right|}^{\left(\left(r_{2}+1\right)/2\right)}+\frac{1}{2}{\bar{\tau }}^{2}\\ +\frac{1}{2}\varepsilon^{2}-\frac{1}{2}\sigma {\tilde{\Theta }}^{T}\tilde{\Theta }+\frac{1}{2}\sigma \Theta^{T}\Theta \\ \leq -\rho V+C, \end{array}$$

where *ρ* and *C* are positive constants defined as

(30) $$\begin{array}{c} \rho =\left\{\frac{2\lambda_{\min}\left(k-I\right)}{\lambda_{\max}\left(M_{0}\right)},\frac{\sigma }{\Gamma^{-1}}\right\},\\ C=\frac{1}{2}{\bar{\tau }}^{2}+\frac{1}{2}\varepsilon^{2}+\frac{1}{2}\sigma \Theta^{T}\Theta . \end{array}$$

To ensure that *ρ* > 0, gains *k* are selected to satisfy

(31) $$\begin{array}{c} \lambda_{\min}\left(k-I\right)>0. \end{array}$$

According to Lemma 2, it can be concluded that *r* and $\tilde{\Theta }$ are bounded. From expression (13), we can infer that*z*_1_ is bounded. Further, based on Lemma 1, it can be concluded that the error of the system is bounded and the output constrains are not violated.

(2) A positive definite Lyapunov function is chosen as

(32) $$\begin{array}{c} V_{2}=\frac{1}{2}rM_{0}r. \end{array}$$

Differentiating (32), we can get

(33) $$\begin{array}{c} {\dot{V}}_{2}=rM_{0}\dot{r}+\frac{1}{2}r{\dot{M}}_{0}r\\ =-kr^{2}-\beta {\text{sig}}^{r_{2}}r^{2}+r\tau_{d}+r\tilde{\Theta }\Phi \left(Z\right)+r\varepsilon \\ \leq -\left(k-\frac{3}{2}I\right)r^{2}-\beta {\left|r^{2}\right|}^{\left(\left(r_{2}+1\right)/2\right)}+\frac{1}{2}{\bar{\tau }}^{2}+\frac{1}{2}\varepsilon^{2}+\frac{1}{2}l^{2}{\tilde{\Theta }}^{2}\\ \leq -\rho_{1}V_{2}-\rho_{2}V_{2}^{\left(\left(r_{2}+1\right)/2\right)}+c, \end{array}$$

where *ρ*_1_, *ρ*_2_, and *c* are positive constants defined as

(34) $$\begin{array}{c} \rho_{1}=\frac{2\lambda_{\min}\left(k-\left(3/2\right)\right)}{\lambda_{\max}\left(M_{0}\right)},\\ \rho_{2}=\beta {\left(\frac{2}{\lambda_{\max}\left(M_{0}\right)}\right)}^{\left(\left(r_{2}+1\right)/2\right)},\\ c=\frac{1}{2}{\bar{\tau }}^{2}+\frac{1}{2}\varepsilon^{2}+\frac{1}{2}l^{2}{\tilde{\Theta }}^{2}. \end{array}$$

Based on Lemma 3, auxiliary variable *r* can converge to the region Ω_*r*_ defined as

(35) $$\begin{array}{c} \Omega_{r}=\left\{r\in R^{n}|r\leq \sqrt{2}Y\right\}, \end{array}$$

where *Y* is defined as

(36) $$\begin{array}{c} Y=\min\left\{{\left(\frac{c/\rho_{1}}{\lambda_{\max}\left(M_{0}\right)}\right)}^{\left(1/2\right)},{\left(\frac{c}{\rho_{1}}\right)}^{\left(1/\left(r_{2}+1\right)\right)}{\left(\lambda_{\max}\left(M_{0}\right)\right)}^{-\left(1/2\right)}\right\}. \end{array}$$

And the upper bound of convergence time is as follows:

(37) $$\begin{array}{c} T_{r}=\frac{2}{\rho_{1}\left(1-r_{2}\right)}\ln\left(\frac{\rho_{1}V_{3}^{1-r_{2}}\left(s\left(0\right)\right)+\rho_{2}}{\rho_{2}}\right). \end{array}$$

Once sliding mode variable reaches the sliding surface *r*=0, (12) can be expressed as

(38) $$\begin{array}{c} {\dot{e}}_{1}=-P_{1}\left(e_{1}\right)e_{1}-k_{1}{\text{sig}}^{a_{2}}e_{1}. \end{array}$$

Another positive Lyapunov function is designed as

(39) $$\begin{array}{c} V=\frac{1}{2}e_{1}^{2}. \end{array}$$

After derivative (39), one has

(40) $$\begin{array}{c} \dot{V}=e_{1}{\dot{e}}_{1}. \end{array}$$

Substituting (38) into (40), we can obtain

(41) $$\begin{array}{c} \dot{V}=e_{1}\left(-P_{1}\left(e_{1}\right)e_{1}-k_{1}{\text{sig}}^{a_{2}}e_{1}\right)\\ =-P_{1}\left(e_{1}\right)e_{1}^{2}-k_{1}{\text{sig}}^{a_{2}}e_{1}^{2}\\ \leq -2\kappa_{1}V-2^{\left(\left(a_{2}+1\right)/2\right)}k_{1}V^{\left(\left(a_{2}+1\right)/2\right)}, \end{array}$$

where *κ*_1_=*λ*_min_*P*_1_(*e*_1_) is a positive constant.

According to Lemma 3, the upper bound of convergence time of error variable *e*_1_ is as follows:

(42) $$\begin{array}{c} T_{e}=\frac{2}{2\kappa_{1}\left(1-a_{2}\right)}\ln\frac{2\kappa_{1}V^{\left(\left(1-a_{2}\right)/2\right)}\left(e_{1}\left(0\right)\right)+2^{\left(\left(a_{2}+1\right)/2\right)}k_{1}}{2^{\left(\left(a_{2}+1\right)/2\right)}k_{1}}. \end{array}$$

Based on (37) and (42), position tracking error converges to neighborhood near the zero point in finite time and convergence time *T* satisfies

(43) $$\begin{array}{c} T\leq T_{e}+T_{r}. \end{array}$$

All the proof has been completed.

### 3.2. Simulation

In this section, to verify the practicability of the presented controller, a 2-DOF robotic manipulator is used for the simulation. The mode matrices are defined as

(44) $$\begin{array}{c} M_{0}\left(q\right)=\left[M_{11},M_{12};M_{21},M_{22}\right],\\ C_{0}\left(q,\dot{q}\right)=\left[C_{11},C_{12};C_{21},0\right],\\ G_{0}\left(q\right)=\left[G_{1};G_{2}\right],\\ \tau_{d}=\left[\tau_{d1},\tau_{d2}\right], \end{array}$$

where *M*_11_=(*m*_1_+*m*_2_)*r*_1_^2^+*m*_2_*r*_2_^2^+2*m*_2_*r*_1_*r*_2_cos(*q*_2_), *M*_22_=*m*_2_*r*_2_^2^, *M*_12_=*M*_21_=*m*_2_*r*_2_^2^+*m*_2_*r*_1_*r*_2_cos(*q*_2_), $C_{11}=-m_{2}r_{1}\sin\left(q_{2}\right){\dot{q}}_{2}$, $C_{12}=-m_{2}r_{1}\sin\left(q_{2}\right)\left({\dot{q}}_{1}+{\dot{q}}_{2}\right)$, *C*_21_=*m*_2_*r*_1_sin(*q*_2_)*q*_1_, *G*_1_=(*m*_1_+*m*_2_)*r*_1_cos(*q*_2_)+*m*_2_*r*_2_cos(*q*_1_+*q*_2_), *G*_2_=*m*_2_*r*_2_cos(*q*_1_+*q*_2_), *τ*_*d*1_=0.5+0.3sin(*t*), and *τ*_*d*2_=0.3+0.5cos(2*t*). Parameters appearing above are shown in Table 1.

Mode uncertainties *M*_*n*_, *C*_*n*_, *G*_*n*_ are set as *M*_*n*_=0.01*M*_0_, *C*_*n*_=0.02*C*_0_, *G*_*n*_=0.01*G*_0_. The initial states $q_{1},q_{2},{\dot{q}}_{1},{\dot{q}}_{2}$ are set as *q*_1_=*q*_2_=0.005 and ${\dot{q}}_{1}={\dot{q}}_{2}=0$. The control goal is to make the output *q* track the target trajectory *q*_1*d*_=*q*_2*d*_=0.3sin(*t*). The output constraints are set as *k*_*o*1_=*k*_*o*2_=0.305.

To verify the validity of the proposed control scheme, there are two controllers that are used as comparison in the following:

1. AFTSM: this is the controller proposed in this paper. The parameters of TSM controller are given as *k*=[20; 20], *k*_1_=[5; 5], *β*=[5; 5], *α*_2_=(5/7), *r*_2_=(7/11). The parameters of error transformation are imposed as *p*_1_=*p*_2_=1. For fuzzy approximator, the initial values of free parameter are all set as 3. The fuzzy learning gain parameters Γ=[10,10], and the adaptive parameter *σ* should be set as a small value [0.01, 0.01], because a large value will suppress the adaptive speed.
2. TSM: this is a general fast terminal sliding mode controller without error transformation and fuzzy approximation. The parameters of TSM controller are given as *k*=[20; 20], *k*_1_=[5; 5], *k*_2_=[6; 6], *β*=[5; 5]*α*_2_=(5/7), *r*_2_=(7/11).

**Remark 3 .**

Sliding mode parameter 0 < *a*_2_ < 1 in (13) will lead to singular problem. So, in the simulation process, use subsection function *φ*(*e*) instead of original sig^*a*_2_^*e*. The subsection function *φ*(*e*) is designed as

(45) $$\begin{array}{c} \varphi \left(e\right)=\left\{\begin{array}{cc} {\left|e\right|}^{a_{2}}\mathrm{sgn}\left(e\right), & s=0\text{ or }s\neq 0,\left|e\right|>\chi ,\\ l_{1}e+l_{2}{\left|e\right|}^{2}\mathrm{sgn}\left(e\right), & s\neq 0,\left|e\right|\leq \chi , \end{array}\right. \end{array}$$

where *χ* is a sufficiently small and bounded positive constant. *a*_2_=(*p*/*q*) is satisfied *p* < *q* and *p* and *q* are coprime positive odd numbers. *l*_1_=(2 − *a*_2_)*χ*^*a*_2_−1^ and *l*_2_=(*a*_2_ − 1)*χ*^*a*_2_−1^.

The simulation results are shown in Figures 4–12.  Figure 4 indicates that the above two control schemes all can track desired trajectory *q*_*d*_. But it can be clearly seen that the AFTSM with error transformation gives smaller error and better tracking performance.  Figure 5 indicates that the tracking errors of proposed controller and TSM all can converge to the neighborhood near the balanced point in finite time. Compared with AFTSM, the convergence rate of TSM is slower than AFTSM, and the transient performances are inferior to AFTSM. Moreover, the output constraints are not limited. The FLS approximation error is shown in Figure 6. It can be seen from the picture that the nonlinear function is well approximated by fuzzy logic system. The norms of fuzzy adaptive weights are shown in Figure 7, from which we can get that the fuzzy weights are bounded.  Figure 8 gives the tracking errors under different initial conditions. From the figure, it can be seen that the convergence time is different for different initial state *q*. The absolute value of the initial state *q* is smaller; the convergence speed is faster.

The discontinuity of sign function sgn(·) can cause system chattering. In order to reduce the chattering of the system, the hyperbolic tangent function *ϖ*(*s*, *ρ*)=((*e*^*ρs*^ − 1)/(*e*^*ρs*^+1)) is used instead of the sign function. By choosing appropriate parameter *ρ*, the chattering phenomenon and the tracking performance of the system can be balanced. Here, choose *ρ* as 2. Comparing Figure 9 with Figure 10, it can be seen that the hyperbolic tangent function can reduce chattering. To verify the robustness of the system to different disturbances, we added three disturbance comparison groups in the simulation. The three groups are set as *d*1=[tan(*t*)+0.7; tan(*t*)+0.7], *d*2=[0.4+2sin(*t*)cos(*t*); 0.2+3sin(*t*)cos(*t*)], $d3=\left[2\sin\left(t\right)q_{1}+{\dot{q}}_{1};3\cos\left(q_{1}\right)+2{\dot{q}}_{1}\right]$. The results are shown in Figure 11; from the picture, one can find that the system still maintains good tracking performance in response to different disturbances.  Figure 12 is the position tracking of step function. The selection of the initial state of the system should ensure that the initial error is satisfied |*e*_1_| < *k*_*b*_. It can be seen from the figure that AFTSM still has a good tracking effect for the step response.

## 4. Conclusions

In this paper, we developed a TSM-based fuzzy adaptive control scheme for robotic manipulators with output constraints and unknown disturbances. An error transformation is used to solve the problems of output constraints. The transient response of the system is improved simultaneously. Fast terminal sliding mode can improve convergence speed and reduce chattering. Therefore, the errors converge to the neighborhood near the balanced point in a very short time. To verify the effectiveness of the proposed scheme, two control schemes are used as a contrast in simulation. The simulation results show that the proposed control method possessed enhanced robustness and better tracking performance.

## Figures and Tables

**Figure 1:** Structure of the fuzzy system.

**Figure 2:** Error transformation.

**Figure 3:** Diagram of the proposed control structure.

**Figure 4:** Position tracking performance of joint 1 and joint 2.

**Figure 5:** Position tracking errors of joint 1 and joint 2.

**Figure 6:** Fuzzy logic system approximate errors.

**Figure 7:** Norms of fuzzy logic weights.

**Figure 8:** Tracking errors under different initial conditions.

**Figure 9:** The inputs in the case of using signum function.

**Figure 10:** The inputs in the case of using hyperbolic tangent function.

**Figure 11:** Position tracking performance under different disturbances.

**Figure 12:** Position tracking performance of step signal.

**Table 1:** Model parameters of the manipulator.

Parameters	Description	Unit	Value
*m*_1_	Mass of link 1	kg	1
*m*_2_	Mass of link 2	kg	1.5
*r*_1_	Length of link 1	m	1
*r*_2_	Length of link 2	m	0.8

## Data Availability

The experiment data used to support this study are available from the corresponding author upon request.
